# Translation Elongation Factor 4 (LepA) Contributes to Tetracycline Susceptibility by Stalling Elongating Ribosomes

This article has been retracted.

**DOI:** 10.1128/AAC.02356-17

**Published:** 2018-07-27

**Authors:** Bin Liu, Chunlai Chen

**Affiliations:** a School of Life Sciences, Tsinghua-Peking Joint Center for Life Sciences, Beijing Advanced Innovation Center for Structural Biology, Tsinghua University, Beijing, China

**Keywords:** elongation factor 4, ribosome profiling, ribosomes, tetracyclines

## Abstract

Even though elongation factor 4 (EF4) is the third most conserved protein in bacteria, its physiological functions remain largely unknown and its proposed molecular mechanisms are conflicting among previous studies. In the present study, we show that the growth of an Escherichia coli strain is more susceptible to tetracycline than its EF4 knockout strain. Consistent with previous studies, our results suggested that EF4 affects ribosome biogenesis when tetracycline is present. Through ribosome profiling analysis, we discovered that EF4 causes 1-nucleotide shifting of ribosomal footprints on mRNA when cells have been exposed to tetracycline. In addition, when tetracycline is present, EF4 inhibits the elongation of protein synthesis, which leads to the accumulation of ribosomes in the early segment of mRNA. Altogether, when cells are exposed to tetracycline, EF4 alters both ribosome biogenesis and the elongation phase of protein synthesis.

## INTRODUCTION

Protein synthesis is a fundamental requirement for all living cells. The process is carried out on the ribosome where the initiation of translation, elongation, termination, and ribosome recycling occur sequentially in a specific order, with the assistance of several protein factors (1, 2). Additional factors such as elongation factor 4 (EF4), elongation factor P (EF-P), alternative ribosome-rescue factor A and B (ArfA and ArfB), and transfer mRNA (tmRNA) are involved in protein synthesis by rescuing stalled or abnormal elongation of ribosomes under stress conditions (3–7). Among these factors, the physiological functions and molecular mechanisms of EF4 are not well understood, and conflicting models have been proposed to detail its various functions (8–11).

EF4 was first reported in 1986 by March and Inouye and named as LepA, as it is the first cistron for most bacteria in the bicistronic leader peptidase operon (12). It is highly conserved in bacteria and shares a high sequence similarity (55 to 68%) among bacterial orthologs (8). In 2006, Qin et al. demonstrated that EF4 could back-translocate the ribosome by moving tRNAs from the E- and P-sites to the P- and A-sites (8) and defined it as an elongation factor. Kinetic studies showed that EF4-induced back-translocation takes several minutes to complete (13). In addition, Liu et al. have shown that during elongation, EF4 competes with elongation factor G (EF-G) to bind to pretranslocation (PRE) ribosomal complexes (9), which raises the question whether back-translocation is the main function of EF4. Results from ribosome profiling suggest that EF4 contributes to the translation initiation and relieves ribosomes paused at glycine codons of several specific genes (10). A recent study proposed that EF4 functions in the biogenesis of the 30S ribosomal subunits because 30S particles accumulate (11). Structures of ribosome-bound EF4 have been visualized with both pretranslocation (PRE) and posttranslocation (POST) ribosomal complexes (14–18). Despite the results from biochemical, cellular, and structural studies, the role of EF4 under stress conditions remains controversial.

EF4 supposedly fulfills its functions under stress conditions as it is located in the membrane under normal growth and is released to the cytosol under certain stress conditions (19). Studies have shown that EF4 accelerates protein synthesis at high Mg^2+^ concentrations (19), low pH (20), and low temperatures (19) and provides a viability advantage for cells under these unfavorable growth conditions. Fredrick and coworkers showed that EF4 contributes to the resistance of Escherichia coli to tellurite, whose cellular toxicity is caused by the oxidization of thiol groups of periplasmic or membrane proteins (21). On the other hand, the deletion of the EF4-encoding gene, *lepA*, could assist the survival of E. coli under several lethal stress conditions (22). In addition, the deletion of *lepA* in Streptomyces coelicolor enhances the production of the calcium-dependent antibiotic (23). Together, these observations suggested that EF4 may have multiple physiological functions.

In the present study, we screened several antibiotics which target the ribosome and inhibit protein synthesis (24). We examined whether they can cause a significant growth differential between an EF4 knockout E. coli strain (JW2553, denoted as the ΔEF4 strain) and its parental strain (BW25113, denoted as the WT strain), both of which were obtained from the Keio collection (25). Among the antibiotics tested, tetracycline was found to be the only one that causes the ΔEF4 strain to grow significantly faster than the WT strain. To understand the effect of EF4 on translation in detail, we performed ribosome profiling and found that the presence of tetracycline resulted in EF4-mediated 1-nucleotide (nt) shifting of ribosomal footprints toward the 5′ end of mRNA and also the accumulation of ribosomes in the early segment of the mRNA open reading frame. Altogether, our results suggested that in the presence of tetracycline, EF4 inhibits protein synthesis by stalling ribosomes in the early elongation cycles.

## RESULTS

### EF4 contributes to tetracycline susceptibility of E. coli.

We tested seven antibiotics that target ribosomes to inhibit protein synthesis via distinctly different mechanisms (see Table S1 in the supplemental material) to carefully examine whether they affect the growth of WT and ΔEF4 strains differently. Tetracycline was the only compound to cause a significant growth differential. The growth of the WT strain was restricted to 50% in the presence of 2.1 ± 0.4 μg/ml tetracycline (the concentration for 50% of maximal growth inhibition [GI_50_]) compared to growth without any antibiotic. When the strain lacked functional EF4, 57 ± 12 μg/ml tetracycline (GI_50_) was required to reduce the overall growth by 50% (Fig. 1a). Thus, in the absence of EF4, cells were less susceptible to tetracycline-induced growth inhibition. This observation is consistent with the previous findings that EF4 promotes cell death under lethal stress conditions (22). Other antibiotics, such as streptomycin, erythromycin, spectinomycin, hygromycin B, puromycin, and gentamicin, inhibited the growth of both strains to similar extents (see Fig. S1). In the ΔEF4 strain, the EF4-encoding gene, *lepA*, was replaced by a kanamycin resistance gene (25), and introducing an empty vector containing the kanamycin resistance gene did not affect the growth of the WT strain in the presence of tetracycline (see Fig. S2). In addition, expression of plasmid-encoded EF4 in the ΔEF4 strain restored its sensitivity to tetracycline (Fig. S2). Altogether, these results indicate that when EF4 is present, E. coli is more susceptible to the effects of tetracycline.

**FIG 1:** EF4 contributes to the growth of E. coli and ribosome biogenesis. (a) Growth of the WT and ΔEF4 strains under different concentrations of tetracycline. Polysome profiles for the WT and ΔEF4 strains without tetracycline treatment (b) and with tetracycline treatment (c). (d) Percentages of subunits (including free 30S and 50S subunits), 70S, and polysomes for the WT and ΔEF4 strains under both tetracycline-treated and untreated conditions.

### Ribosome biogenesis is affected in the WT strain under tetracycline stress.

Next, we found that ribosomal subunits were aberrantly accumulated in the WT strain under tetracycline stress, whereas no such accumulation of ribosomal subunits was found in the ΔEF4 strain with tetracycline and in both strains, WT and ΔEF4, without tetracycline (Fig. 1b to d). To carefully examine these accumulated subunit fractions, we optimized the experimental conditions for sucrose gradient ultracentrifugation to separate these fractions (see Fig. S3). Three peaks containing ribosomal subunits were obtained for the WT strain under tetracycline stress. After examining proteins in each peak via SDS-PAGE, two of them were assigned as fractions of ribosomal 30S subunit and one of them was assigned to the fraction of ribosomal 50S subunit. Clearly, one of 30S subunit fractions was immature, as previously reported (11), because it lacked most of the ribosomal proteins located on the 30S subunit (Fig. S3c). From our experiments, we could not resolve whether other 30S and 50S fractions were mature or not. In all, we observed that ribosome biogenesis is affected in the WT strain under tetracycline stress.

Interestingly, we found that *rpsN* (ribosomal protein S14) and *rpsU* (ribosomal protein S21) were significantly downregulated at the translational level in the ΔEF4 strain (Fig. S4), which agrees with a previous report that in the ΔEF4 strain, these two ribosomal proteins were absent in a small portion of 30S subunits (11). Upon treatment of WT and ΔEF4 strains with tetracycline, we observed that most ribosomal proteins were significantly downregulated in the ΔEF4 strain at both translational and transcriptional levels (Fig. S4). On the other hand, *rmf*, *sra*, *hpf*, and *lysU* were significantly upregulated in the ΔEF4 strain at both translational and transcriptional levels.

### EF4 causes 1-nt shifting of ribosomal footprints with tetracycline.

In our study, the length distributions of ribosomal footprints peaked at 26 nt for all samples (Fig. 2a). We selected 20- to 36-nt-length footprints for further analysis. To identify the location of the P-site on ribosomal footprints, we created a profile of the 5′-end positions of reads as a function of the distance from the start codon of their genes and a profile of 3′-end positions of reads as a function of the distance from the stop codons of their genes (Fig. 2b to f), which were used to determine the distances of the ribosomal P-site from the 5′ end and the 3′ end of the footprints, respectively. Consistent with a previous report (26), the distances between the P-site and the 3′ end of the footprints remained mostly the same for footprints of different lengths, whereas the distances between the P-site and 5′ end of the footprints decreased linearly when the lengths of the footprints decreased (Fig. 2c to f). In the absence of tetracycline, the locations of the P-site on ribosomal footprints were the same for both WT and ΔEF4 strains (Fig. 2c and d). However, in the presence of tetracycline, the locations of the P-site on footprints had a 1-nt difference between WT and ΔEF4 strains (Fig. 2e and f). These results indicate that in WT cells treated with tetracycline, EF4 causes a 1-nt shift of ribosomal footprints toward the 5′ end of mRNA.

**FIG 2:** Ribosomal footprints analysis. (a) Length distributions of ribosomal footprints for four samples. (b) The plot shows how P-site offsets could be determined from the distribution of distances from the 5′ end of the footprints to the start codon and distribution of distances from 3′ end of footprints to the stop codon. Plots of footprint length versus the offsets between the 5′ end and the start codon for the untreated (c) and tetracycline-treated (e) samples. The *x* axes show the nucleotide positions upstream of the start codon. Plots of footprint length versus the offsets between 3′ end and stop codon for the untreated (d) and tetracycline-treated (f) samples. The *x* axes show the nucleotide positions downstream of the stop codon. (g) Schematic demonstrates that EF4 causes 1-nt shifting of ribosomal footprints toward the 5′ end of mRNA.

### EF4 causes accumulation of ribosomes in the early segment of mRNAs under tetracycline treatment.

We noticed that in the presence of tetracycline, ribosomal footprints of the WT strain accumulated in the early segment of mRNAs, whereas ribosomal footprints were distributed more evenly under the other three conditions (Fig. 3a and b; see also Fig. S5). Such phenomena can be verified by examining the ratios between the number of ribosomal footprints on the first half of each mRNA and the number of footprints on the second half (Fig. 3c to f). Clearly, for the WT strain upon treatment with tetracycline, there were more mRNAs with ribosomes accumulated in the first half of the transcripts. In addition, during the preparation of ribosomal footprints, we observed that only dimeric and trimeric ribosomes were present in the tetracycline-treated WT strain after polysomes were subjected to mRNA digestion by micrococcal nuclease (MNase) (Fig. 3g). For these undigested dimeric and trimeric ribosomes, mRNA fragments were likely to be protected from MNase digestion by the clustering of nearby ribosomes, which were close to each other, preventing the MNase from accessing the mRNA. Similar phenomena have been reported elsewhere (27, 28). In addition, we found that the average ribosome density (ARD) was higher in the WT strain after tetracycline treatment, whereas the ARDs in WT and ΔEF4 strains were similar under normal conditions (Fig. 3h and i). There was a significant accumulation of ribosomes at the start codon after tetracycline treatment (Fig. 3j and k). These results suggest that the decreased viability of the WT strain under tetracycline stress is not due to fewer ribosomes on the mRNA but to ribosome stalling during elongation. Altogether, our findings indicate that in the presence of tetracycline, EF4 severely inhibits the elongation phase of protein synthesis and causes an accumulation of ribosomes in the early segment of transcripts and “traffic jams” of ribosomes.

**FIG 3:** EF4 mediates ribosome stalling during elongation under tetracycline stress. Profiles of ribosomal footprints on mRNA of gene *gapA* in the WT (a) and ΔEF4 (b) strains with tetracycline treatment. The scatter plots of total number of footprints (*y* axis) versus ratio between the number of footprints on the first half and on the second half of mRNA (*x* axis) for all the genes in the WT (c) and ΔEF4 (d) strains without tetracycline treatment and in the WT (e) and ΔEF4 (f) strains with tetracycline treatment. (g) The polysomal profiles after MNase digestion. Dimeric and trimeric ribosomes were present in the WT strain. Changes of average ribosome density (ARD) between the WT and ΔEF4 strains in the absence (h) or presence (i) of tetracycline. ARD around the start codon (defined as 0) in the absence (j) or presence (k) of tetracycline.

### EF4 mediates ribosome stalling at specific codons under tetracycline stress.

To determine whether ribosomes are stalled at specific codons, we calculated the frequencies of 61 codons at the ribosomal A-, P-, and E-sites using Ribo-seq unit step transformation (RUST) software (29). Consistent with a previous study (10), the frequencies of glycine codons (GGC and GGT) were higher in the ΔEF4 strain than in the WT strain at the ribosomal A- and P-sites (Fig. 4a and b). Interestingly, we observed that in the presence of tetracycline, the frequencies of arginine (AGG, CGG, CGA, and AGA), serine (TCG, AGT, and AGC), and threonine (ACG and ACA) codons were higher in the WT strain than the ΔEF4 strain (Fig. 4; see also Fig. S6). Previous studies have shown that EF4 can interact with the peptidyl transferase center and tRNA through its C-terminal domain (14–16). Therefore, we speculated that arginine, serine, and threonine residues might interact with EF4's C-terminal domain through their side chains and cause significant ribosome stalling and high resident frequencies on these codons in the presence of tetracycline.

**FIG 4:** Ribosome stalling on specific codons. RUST ratios of several codons at A-sites (a), P-sites (b), and E-sites (c) for all four samples.

## DISCUSSION

EF4 is the third most conserved protein in bacteria (8) and commonly known to have three major functions, which are to promote back-translocation, to sequester elongating ribosomes, and to assist in 30S subunit biogenesis. EF4 behaves as a bifunctional factor in a cellular stress response that promotes cell survival or cell death, depending on the severity of the stress. Results from structural (14–18), biochemical (9, 11), and cellular (10) studies led to conflicting models to interpret EF4 functions. Therefore, the discovery of novel EF4-mediated cellular phenotypes is an alternative approach to reveal its functions. In this study, we screened several antibiotics that are known to target the ribosomes and inhibit protein synthesis via different mechanisms. We discovered that tetracycline causes a growth differential between the WT and ΔEF4 E. coli strains. Our results from ribosome profiling support the model that EF4 contributes to both ribosome biogenesis and ribosome stalling during the elongation phase of protein synthesis under tetracycline stress.

Previous studies have suggested that EF4 mediates the biogenesis of ribosomal 30S subunits. By using stable isotope labeling using amino acids in cell culture-mass spectrometry (SILAC-MS), Fredrick and colleagues found that 30S subunits lacking S3, S10, S14, and S21 proteins are accumulated in the cells in the absence of EF4 (11). Under tetracycline stress, we also found that the expression levels of S14 and S21 were significantly lower in the ΔEF4 strain than in the WT strain. In general, our results supported the model that EF4 contributes to ribosome biogenesis. On the other hand, upon treatment with tetracycline, ribosomal subunits only abnormally accumulated in the WT strain (Fig. 1c). The accumulation of ribosomal subunits may be due to stalled ribosomes located at and around the start codon (Fig. 3k), which prevents further initiation and formation of 70S on the mRNA from separated ribosomal subunits. In addition, the presence of immature 30S subunits (Fig. S3 in the supplemental material) indicated a subunit assembly defect. Altogether, we discovered that EF4 is likely to affect ribosome biogenesis and 70S assembly, through both direct and indirect pathways, under tetracycline stress.

Tetracycline is known to interact with 16S rRNAs, including C1054 in h34, and to inhibit protein synthesis by preventing the attachment of aminoacyl-tRNA to the ribosomal A-site (30, 31). Therefore, tetracycline is likely to stall ribosomes in their POST states containing an empty A-site (32). Recently, using single-molecule fluorescence resonance energy transfer assays, we discovered that EF4 interacts with both ribosomal PRE and POST complexes (33). Interactions between EF4 and the PRE complex accelerate translocation, which leads to the formation of the POST complex. On the other hand, interactions between EF4 and the POST complex impair the delivery of aminoacyl-tRNA into the A-site of the ribosome. Therefore, EF4 would mainly stall ribosomes in their POST state (33), which is more accessible for tetracycline binding than the PRE complex. Altogether with the previous reports and the results observed in this study, we hypothesize that EF4 might interact with tetracycline-stalled POST complexes to further enhance the stalling effect caused by tetracycline. The fact that EF4 caused 1-nt shifting of ribosomal footprints with tetracycline suggests that EF4 might interact with tetracycline-stalled ribosomes in cells to modulate the conformation of the ribosomes. Although tetracycline alone could cause a decrease in the polysome fractions and an accumulation of ribosomes around the start codons, EF4 further increased the 30S and 50S fractions and enhanced the accumulation of ribosomes around the start codons (Fig. 1d and 3k). Such phenomena supported our hypothesis that an interaction between EF4 and a tetracycline-stalled ribosomal complex can further enhance the stalling effect. We speculate that all the other antibiotics we used (Table S1), except tetracycline, target the ribosomal complexes and translation steps which cannot interact with or be effectively modulated by EF4. Therefore, no other antibiotics caused a significant growth differential between the WT and ΔEF4 strains. In conclusion, we discovered that EF4 directly interacts with ribosomes to inhibit elongation under tetracycline stress.

Major mechanisms of resistance to tetracycline include mutations in tetracycline binding sites (34), tetracycline-specific ribosomal protection (35–37), tetracycline-specific efflux (38, 39), and tetracycline inactivation by enzymes (40). To the best of our knowledge, for the first time, we discovered that EF4 contributes to the tetracycline susceptibility of E. coli cells (27-fold increase of GI_50_). Our results suggest that EF4, directly and indirectly, affects the maturation and assembly of the ribosome under tetracycline stress. Furthermore, our studies revealed that EF4 mediates global ribosome stalling and causes an accumulation of ribosomes in the early segments of mRNAs under tetracycline stress. All the data presented in this study support the model that EF4 affects ribosome biogenesis and stalls elongating ribosomes to inhibit global protein translation, which eventually contributes to tetracycline susceptibility.

## MATERIALS AND METHODS

### Antibiotic screening and bacterial culture.

The EF4 knockout E. coli strain (JW2553, denoted the ΔEF4 strain) and its parental strain (BW25113, denoted the WT strain) were obtained from the Keio collection (25). The genotypes of the WT and ΔEF4 strains were ′*rrnB3* Δ*lacZ4787 hsdR514* Δ(*araBAD*)*567* Δ(*rhaBAD*)*568 rph1*′ and ′*rrnB3* Δ*lacZ4787 hsdR514* ΔEF4::Km Δ(*araBAD*)*567* Δ(*rhaBAD*)*568 rph1*′, respectively. Both strains were cultured in Luria-Bertani (LB) medium overnight at 37°C in a shaker. Then they were diluted in LB medium to an optical density at 600 nm (OD_600_) of 0.05 and shaken at 37°C for another 7 h with or without antibiotics. Each experiment was done in triplicates. Three identical replicates were performed in parallel each time. We estimated the concentration for 50% of maximal growth inhibition (GI_50_) as the concentration of tetracycline at which the final OD_600_ is 50% of the final OD_600_ in the absence of tetracycline.

### Polysome extraction, ultracentrifugation, and mRNA isolation.

Both WT and ΔEF4 strains were cultured in 200 ml LB medium containing 4 μg/ml tetracycline hydrochloride at 37°C and harvested at an OD_600_ of ∼0.30. In the absence of tetracycline, cells were harvested at an OD_600_ of ∼0.40. Equal volumes of ice were added to the harvested cells and mixed immediately. The mixtures were centrifuged at 5,000 rpm for 6 min at 4°C (TX-400 swinging bucket rotor; Thermo Scientific). The pellets obtained were resuspended in 650 μl lysis buffer containing 10 mM MgCl_2_, 100 mM NH_4_Cl, 20 mM Tris (pH 8.0), 1 mg/ml lysozyme (L8120; Solarbio), 100 U/ml of RNase-free DNase I (EN0521; Thermo Scientific), and 0.5 U/μl of Superase·In (AM2696; Invitrogen) and subjected to three freeze-thaw cycles. Sodium deoxycholate was added to the solutions to a final concentration of 0.1% (wt/vol). The lysates were incubated on ice for 10 min and centrifuged at 12,000 rpm for 10 min to obtain the supernatants containing polysomes. Each of the supernatants was aliquoted into three RNase-free tubes; one of them was utilized to construct the ribosome profiling sequencing library, one was utilized to perform polysome analysis through sucrose gradient ultracentrifugation, and the other was used to isolate mRNA with TRIzol reagent (Invitrogen) according to the manufacturer's protocol. Total mRNAs were fragmented by alkaline hydrolysis, and ∼300-bp-length fragments were picked from an SDS-PAGE gel to generate a cDNA library according to a published procedure (41).

Sucrose gradient ultracentrifugation experiments were conducted by loading 10 *A*_260_ units of supernatant onto a 10 to 50% sucrose gradient in buffer (10 mM MgCl_2_, 100 mM NH_4_Cl, 20 mM Tris [pH 8.0], and 2 mM dithiothreitol [DTT]) and centrifuging for 2.5 h at 40,000 rpm in a Beckman rotor (SW-41). Gradients were fractionated using a Brandel density gradient fractionator equipped with a UV absorbance detector.

### Ribo-seq library construction.

Ribo-seq libraries were constructed according to the published protocols with minor modifications (42–44). In brief, 25 *A*_260_ units of clarified lysate were cleaved with 1,200 units of MNase (Sigma, Roche) into monosomes (70S ribosome), which were then separated and collected through sucrose gradient ultracentrifugation. Ribosome-protected footprint fragments were extracted with an miRNeasy minikit (Qiagen). Fragments between 15 and 45 nt in length were picked via denaturing urea-polyacrylamide gel electrophoresis. A linker (New England BioLabs) was ligated onto purified RNA fragments. Then, a reverse transcription reaction (Invitrogen) was conducted to generate cDNAs, which were circulated with CircLigase (Epicentre). Biotinylated DNA oligonucleotides (see Table S2 in the supplemental material) were mixed at a concentration of 10 μM each to hybridize with circulated cDNAs at 37°C for 15 min in a ThermoMixer (Eppendorf) and were removed via streptavidin affinity. Finally, a Ribo-seq library was generated by PCR with high-fidelity Phusion DNA polymerase (New England BioLabs). All the primers used for reverse transcription and PCR amplification are listed in Table S2. 5′-End biotinylated DNA oligonucleotides were designed to complement reads of rRNAs in published data (10).

### Sequencing.

Ribo-seq libraries and mRNA libraries were loaded into two lanes of an Illumina HiSeq 2500 sequencer to generate approximately 2 GB raw data for each library.

### Read quality control and adapter trimming.

Any reads with a Phred quality score below 20 (99% base call accuracy) were removed. Adapters of the ribosome protected fragments were cut with cutadapt software (version 1.14) with default parameters. Finally, reads shorter than 20 nt or longer than 36 nt were discarded with cutadapt software (45).

### Read alignment.

The Ribo-seq reads and mRNA reads were mapped to the BW25113 genome (NCBI reference sequence NZ_CP009273.1) by using bowtie2 (version 2.2.9) with default parameters (46). On the basis of the default settings of bowtie2 software, one location was chosen randomly from the possible mapping sites for further analysis of the multiply aligned reads. The sam files were converted to bam format, sorted, and indexed using Samtools (version 0.1.19) (47).

### P-site determination.

A previous study showed that the distance between the 3′ end of ribosome footprint reads and the P-site is less variable than the distance between the 5′ end of reads and the P-site (26). Hence, we performed a metagene analysis of the 3′-end position of each length of reads around the stop codon with Plastid software (48) using combined data from two replicates. For most read lengths, this analysis shows a peak located 15 nt downstream from the first nucleotide of the stop codon for WT and ΔEF4 strains and the ΔEF4 strain treated with tetracycline and a peak located 14 nt downstream for the WT strain treated with tetracycline. Several references indicate that these peaks are associated with a termination of translation (44, 49). Therefore, we assigned 16 nt as the offset of the P-site from the 3′ ends of reads for WT and ΔEF4 strains and the ΔEF4 strain treated with tetracycline and 15 nt for the WT strain treated with tetracycline. We also determined the P-site offsets from 5′ ends of reads around the start codon using psite script in Plastid software (48).

### Calculation of average ribosome density.

We used the P-site offset to assign a position on mRNAs for each read. The total number of reads was summed at each nucleotide position for all mRNAs. The average ribosome density (ARD) was obtained using the total number of reads at each position divided by the total number of genes. The ARD obtained was normalized by dividing by the total number of reads of the sample.

### Ribo-seq unit step transformation analysis.

Ribo-seq unit step transformation (RUST) written by Baranov and coworkers was used to process the ribosome profiling data (29). The predominant length of reads was subjected to RUST analysis at RiboGalaxy (http://ribogalaxy.ucc.ie). The RUST ratios of codons at ribosomal A-, P-, and E-sites were determined according to the guidance of the program.

### Differentially expressed gene analysis.

Counts of reads for each gene were calculated using Plastid (48) with the corresponding offset and the midpoint of reads in mRNA sequencing data. The significance test was implemented using DEseq2 software (50).

### Statistical tests.

All statistical tests were performed using the R statistical programming package version 3.4.0. The correlations of replicates for all samples are shown in Fig. S7 in the supplemental material.

### Accession number(s).

Sequencing data were deposited at the NCBI Gene Expression Omnibus under study accession number GSE106448.

## Supplementary Material

Supplemental file 1
